# Earnings Management Behavior of Enterprise Managers Based on Evolutionary Game Theory

**DOI:** 10.1155/2022/8037226

**Published:** 2022-03-19

**Authors:** Yang Wang, Anqi Li, Jiahuan Liu

**Affiliations:** China University of Mining and Technology, Beijing 100083, China

## Abstract

Today, earnings mismanagement in China's enterprises has become a serious problem as managers conduct financial fraud by means of earnings management, hindering China's overall economic development. Upon shareholders' requirements and investors' concerns, managers should disclose real financial information. The essay analyzes the revenue function generated by the manager and the shareholder through an evolutionary theory model where the managers team of the enterprise and shareholders are both game parties. After building the model, the essay utilizes Python to stimulate the theoretical model to analyze both parties' behavior to explain the process of evolutionary game theory.

## 1. Introduction

For decades, enterprise managers misusing earnings management for personal interests have been headlines. Financial fraud has become one of the key issues discussed in relevant circles for theoretical and practical perspectives. Many enterprises create fake profits by manipulating earnings management to mislead investors who may invest more in the company once they believe its good performance. Meanwhile, there are some enterprises that modify the financial reports with a shrunk profit to avoid tax by increasing the cost expenses of the company, etc. [1–4]. Against such a context, it is necessary to study enterprise earnings management. Schipper believes that earnings management is a purposeful intervention in the external financial reporting process, with the intent of obtaining some private gain managers [5]. As Canadian scholar Scott writes in his work, earnings management is defined as the choice by enterprise managers who use selected accounting policy to smooth their compensation or maximize the enterprise market value [6]. Liang and Wang established an evolutionary game theory model of PPP projects to study the game pattern of government and private investors, based on which they give specific suggestions [7]. Based on the bounded rational person, Zhang constructed an evolutionary game model to study the sci-tech innovation behaviors of government and small and medium-sized enterprises as the parties of the game.

The paper built an evolutionary game model for managers and the shareholders based on the analysis of relevant variables of both parties to depict the dynamic evolution process of behaviors managers, the decision-making process, and the final stable state displayed by managers and the shareholders. The paper utilizes Python to conduct numerical simulation on the evolution process to show the evolutionary game process of both parties in a more intuitive way.

## 2. Construction of the Game Model of the Manager and Shareholder

The evolutionary game model in this paper is based on the following hypotheses.

**Hypothesis 1 .**

In evolutionary game theory, the game players are managers and shareholders, and both of them are bounded rational persons.

**Hypothesis 2 .**

Both parties of the game adjust their own decisions after examining the decisions made by the other party. As the decision-making behaviors of both parties do not take place simultaneously, this type of game is a dynamic game.

The paper sets managers as Player 1, whose game strategies include have earnings management and no earnings management; and shareholders as Player 2, whose game strategy includes having supervision and no supervision. Assume that the proportion of managers having earnings management is *x*, while the proportion of managers choosing no earnings management is 1 − *x*, in which *x* is the function *x*(*t*) of time *t*. Assume that the probability of supervision by shareholders is *y*, while the probability of no supervision is 1 − *y*, in which *y* is the function *y*(*t*) of time *t*. Assume that the total income of the company is *s*=*s*_1_+*s*_*n*_, and the income *s*_1_ without manager's earnings management is proportional to the total income *s*, namely *s*_1_=*m∗s*=*m∗*(*s*_1_+*s*_*n*_).

The relevant variables in this paper are shown in Table 1, and the payment matrices are shown in Table 2.

From managers' perspective, the earnings management cost paid by managers has effects on the current payment period only, which means that the earnings management cost managers have no cumulative utility and no aftereffect. Assume counterfeiting efficiency as shown in formula (1), which *n*_*c*_2__^*∗*^, *α*_*c*_2__^*∗*^ represents the strength of managers' counterfeiting ability [8–10].

(1) $$\begin{array}{c} a=\overset{*}{\underset{c_{2}}{n}}c_{2\left(t\right)}^{\overset{*}{\underset{c_{2}}{\alpha }}},\alpha >0. \end{array}$$

From the shareholders' perspective, the supervision cost of shareholders in the current period may also influence the identification of the next period, thus showing a cumulative utility. Assuming the expression of supervision efficiency is as shown in formula (2), *n*_*c*_1__^*∗*^, *α*_*c*_1__^*∗*^ represents the degree of shareholders' supervision.

(2) $$\begin{array}{c} b=\overset{*}{\underset{c_{1}}{n}}{\left[\sum_{j=1}^{t}c_{1\left(j\right)}^{*}\right]}^{\overset{*}{\underset{C_{1}}{\alpha }}}. \end{array}$$

Assume the expression of shareholders' supervision cost is as shown in

(3) $$\begin{array}{c} C_{1\left(t\right)}=\sum_{j=t}^{t}\left(c_{1\left(j\right)}^{*}\right). \end{array}$$

Assume the expression of managers' earnings management cost is as shown in

(4) $$\begin{array}{c} C_{2\left(t\right)}={\left[\frac{a}{n_{C_{2}}^{*}}\right]}^{1/\overset{*}{\underset{C_{2}}{\alpha }}}. \end{array}$$

Assume the expression of managers' earnings management cost is as shown in

(5) $$\begin{array}{c} C_{1\left(t\right)}={\left[\frac{b}{n_{C_{1}}^{*}}\right]}^{1/\overset{*}{\underset{C_{1}}{\alpha }}}. \end{array}$$

Assume the expression of shareholders' identification probability is as shown in

(6) $$\begin{array}{c} \beta =1-e^{-b/a}. \end{array}$$

## 3. Evolutionary Game Analysis

### 3.1. Evolutionary Equilibrium Point

According to the above payment matrices, when managers Player 1 chooses earnings management, the expected income and group average income are as shown in formula (7), while no earnings management is shown in formula (8) [11, 12]:

The expected income of managers choosing earnings management is shown as follows:

(7) $$\begin{array}{c} U_{11}=y\left[\frac{m\times s_{n}\left(t\right)}{1-m}+\Delta s\left(t\right)-{\left(\frac{a}{n_{C_{2}}^{*}}\right)}^{1/\overset{*}{\underset{C_{2}}{\alpha }}}-k\left(1-e^{-b/a}\right)\times \Delta s\left(t\right)-d\right]+\left(1-y\right)\\ \times \left[\frac{m\times s_{n}\left(t\right)}{1-m}+\Delta s\left(t\right)-{\left(\frac{a}{n_{C_{2}}^{*}}\right)}^{1/\overset{*}{\underset{C_{2}}{\alpha }}}-d\right]. \end{array}$$

The expected income of the managers choosing no earnings management is shown as follows:

(8) $$\begin{array}{c} U_{12}=y\times \left[\frac{m\times s_{n}\left(t\right)}{1-m}-d\right]+\left(1-y\right)\times \left[\frac{m\times s_{n}\left(t\right)}{1-m}-d\right]. \end{array}$$

Under the above two conditions, the group average income is shown in

(9) $$\begin{array}{c} \bar{U_{1}}=xy\times \left[\frac{m\times s_{n}\left(t\right)}{1-m}+\Delta s\left(t\right)-{\left(\frac{a}{n_{C_{2}}^{*}}\right)}^{1/\overset{*}{\underset{C_{2}}{\alpha }}}-k\left(1-e^{-b/a}\right)\times \Delta s\left(t\right)-d\right]+x\left(1-y\right)\\ \times \left[\frac{m\times s_{n}\left(t\right)}{1-m}+\Delta s\left(t\right)-{\left(\frac{a}{n_{C_{2}}^{*}}\right)}^{1/\overset{*}{\underset{C_{2}}{\alpha }}}-d\right]+\left(1-x\right)\left[\frac{m\times s_{n}\left(t\right)}{1-m}-d\right]. \end{array}$$

When Player 2 chooses supervision, the expected income and group average income are shown in formula (10), while the expected income and group average income are shown in formula (11) when there is no supervision.

The expected income when shareholders supervise is as follows:

(10) $$\begin{array}{c} U_{21}=x\left[s_{n}\left(t\right)-{\left(\frac{b}{n_{C_{1}}^{*}}\right)}^{1/\overset{*}{\underset{C_{1}}{\alpha }}}+k\left(1-e^{-b/a}\right)\Delta s\left(t\right)-\Delta s\left(t\right)\right]+\left(1-x\right)\left[s_{n}\left(t\right)-{\left(\frac{b}{n_{C_{1}}^{*}}\right)}^{1/\overset{*}{\underset{C_{1}}{\alpha }}}\right]. \end{array}$$

The expected income when shareholders do not supervise is shown as follows:

(11) $$\begin{array}{c} U_{22}=x\left[s_{n}\left(t\right)-\Delta s\left(t\right)\right]+\left(1-x\right)\times s_{n}\left(t\right). \end{array}$$

Under the above two conditions, the group average income is as shown in

(12) $$\begin{array}{c} \bar{U_{2}}=xy\left[s_{n}\left(t\right)-{\left(\frac{b}{n_{C_{1}}^{*}}\right)}^{1/\overset{*}{\underset{C_{1}}{\alpha }}}+k\left(1-e^{-b/a}\right)\times \Delta s\left(t\right)-\Delta s\left(t\right)\right]+y\left(1-x\right)\left[s_{n}\left(t\right)-{\left(\frac{b}{n_{C_{1}}^{*}}\right)}^{1/\overset{*}{\underset{C_{1}}{\alpha }}}\right]\\ -x\left(1-y\right)\times \Delta s\left(t\right)+\left(1-y\right)s_{n}\left(t\right). \end{array}$$

According to the above formula, the replicated dynamic equation of managers as Player 1 is figured [13] as shown in

(13) $$\begin{array}{c} F\left(x\right)=\frac{dx}{dt}=x\times \left(U_{11}-{\bar{U}}_{1}\right)=x\left(1-x\right)\left[\Delta s\left(t\right)-{\left(\frac{a}{n_{C_{2}}^{*}}\right)}^{1/\overset{*}{\underset{C_{2}}{\alpha }}}--yk\left(1-e^{-b/a}\right)\times \Delta s\left(t\right)\right]. \end{array}$$

Make *F*(*x*)=0:

(14) $$\begin{array}{c} x_{1}=0,x_{2}=1,y_{3}=\frac{\Delta s\left(t\right)-{\left(a/n_{C_{2}}^{*}\right)}^{1/\alpha_{C_{2}}^{*}}}{k\left(1-e^{-b/a}\right)\Delta s\left(t\right)}. \end{array}$$

According to the previous formula, the replicated dynamic equation of shareholders as Player 1 is figured as shown in [14]

(15) $$\begin{array}{c} F\left(y\right)=\frac{dy}{dt}=y\left(U_{21}-{\bar{U}}_{2}\right)=y\left(1-y\right)\left[xk\left(1-e^{-b/a}\right)\times \Delta s\left(t\right)-{\left(\frac{b}{n_{C_{1}}^{*}}\right)}^{1/\overset{*}{\underset{C_{1}}{\alpha }}}\right]. \end{array}$$

Make *F*(*y*)=0:

(16) $$\begin{array}{c} y_{1}=0,y_{2}=1,x_{3}=\frac{{\left(b/n_{C_{1}}^{*}\right)}^{1/\alpha_{C_{1}}^{*}}}{k\left(1-e^{-b/a}\right)\times \Delta s\left(t\right)}. \end{array}$$

The strategy combination corresponding to the equilibrium point of the replicated dynamic system is an equilibrium point of the evolutionary game or evolutionary equilibrium point for short. According to the above calculations, the paper found five kinds of equilibrium solutions. The equilibrium solutions of (*x*, *y*) are (0, 0) (0, 1) (1, 0) (1, 1) (*x*3, *y*3).

### 3.2. Stability Analysis of Equilibrium Point

The equilibrium points in the evolutionary game can be calculated through the local stability of the Jacobian matrix to analyze the stability of each equilibrium point. According to the Jacobian matrix of the group average income function of both parties in the game shown above, taking the derivative of $\bar{U}1\cdot \bar{U}2$ in turn to obtain the differentials with respect to *x* and *y* will build the Jacobian matrix.

(17) $$\begin{array}{c} \left[\begin{array}{cc} B_{11} & B_{12}\\ B_{21} & B_{22} \end{array}\right], \end{array}$$

where

(18) $$\begin{array}{c} B_{11}=\left(1-2x\right)\left[\Delta s\left(t\right)-{\left(\frac{a}{n_{C_{2}}^{*}}\right)}^{1/\overset{*}{\underset{C_{2}}{\alpha }}}-yk\left(1-e^{-b/a}\right)\Delta s\left(t\right)\right]\\ B_{12}=-x\left(1-x\right)*k\left(1-e^{-b/a}\right)\Delta s\left(t\right)\\ B_{21}=y\left(1-y\right)*k\left(1-e^{-b/a}\right)*\Delta s\left(t\right)\\ B_{22}=\left(1-2y\right)\left[xk\left(1-e^{-b/a}\right)*\Delta s\left(t\right)-{\left(\frac{b}{n_{C_{1}}^{*}}\right)}^{1/\overset{*}{\underset{C_{1}}{\alpha }}}\right]. \end{array}$$

According to the Lyapunov stability theorem, when all eigenvalues of a matrix are negative real numbers, the point has stability; i.e., it is an evolutionary stable point. As *de*  *J*=*λ*_1_+*λ*_2_ (*λ*_1_ and *λ*_2_ are the two eigenvalues of the matrix), and *trJ*=*λ*_1_*∗λ*_2_, *λ*_1_ and *λ*_2_ will be negative numbers only when *de*  *J* > 0 and *trJ* < 0, and the equilibrium point at this time is the evolutionary stable point (*ESS*) of the system [11]:

(1) When *x*, *y* is (0, 0), formula (19) is
  (19) $$\begin{array}{c} \det J=-{\left(\frac{b}{n_{C_{1}}^{*}}\right)}^{1/\overset{*}{\underset{C_{1}}{\alpha }}}\left[\Delta s\left(t\right)-{\left(\frac{a}{n_{C_{2}}^{*}}\right)}^{1/\overset{*}{\underset{C_{2}}{\alpha }}}\right],\\ trJ=-{\left(\frac{b}{n_{C_{1}}^{*}}\right)}^{1/\overset{*}{\underset{C_{1}}{\alpha }}}+\left[\Delta s\left(t\right)-{\left(\frac{a}{n_{C_{2}}^{*}}\right)}^{1/\overset{*}{\underset{C_{2}}{\alpha }}}\right]. \end{array}$$
(2) When *x*, *y* is (0, 1), formula (20) is:
  (20) $$\begin{array}{c} \det J={\left(\frac{b}{n_{C_{1}}^{*}}\right)}^{1/\overset{*}{\underset{C_{1}}{\alpha }}}\left[\Delta s\left(t\right)-{\left(\frac{a}{n_{C_{2}}^{*}}\right)}^{1/\overset{*}{\underset{C_{2}}{\alpha }}}-k\left(1-e^{-b/a}\right)\Delta s\left(t\right)\right],\\ trJ={\left(\frac{b}{n_{C_{1}}^{*}}\right)}^{1/\overset{*}{\underset{C_{1}}{\alpha }}}+\left[\Delta s\left(t\right)-{\left(\frac{a}{n_{C_{2}}^{*}}\right)}^{1/\overset{*}{\underset{C_{2}}{\alpha }}}-k\left(1-e^{-b/a}\right)\Delta s\left(t\right)\right]. \end{array}$$
(3) When *x*, *y* is (1, 0), formula (21) is
  (21) $$\begin{array}{c} \det J=-\left[k\left(1-e^{-b/a}\right)\Delta s\left(t\right)-{\left(\frac{b}{n_{C_{1}}^{*}}\right)}^{1/\overset{*}{\underset{C_{1}}{n}}}\right]\times \left[\Delta s\left(t\right)-{\left(\frac{a}{n_{C_{2}}^{*}}\right)}^{1/\overset{*}{\underset{C_{2}}{n}}}\right],\\ trJ=\left[k\left(1-e^{-b/a}\right)\Delta s\left(t\right)-{\left(\frac{b}{n_{C_{1}}^{*}}\right)}^{1/\overset{*}{\underset{C_{1}}{n}}}\right]-\left[\Delta s\left(t\right)-{\left(\frac{a}{n_{C_{2}}^{*}}\right)}^{1/\overset{*}{\underset{C_{2}}{n}}}\right]. \end{array}$$
(4) When *x*, *y* is (1, 1), formula (22) is
  (22) $$\begin{array}{c} \det J=\left[k\left(1-e^{-b/a}\right)\Delta s\left(t\right)-{\left(\frac{a}{n_{C_{2}}^{*}}\right)}^{1/\overset{*}{\underset{C_{2}}{\alpha }}}\right]\times \left[\Delta s\left(t\right)-{\left(\frac{a}{n_{C_{2}}^{*}}\right)}^{1/\overset{*}{\underset{C_{2}}{\alpha }}}-k\left(1-e^{-b/a}\right)\Delta s\left(t\right)\right],\\ trJ={\left(\frac{b}{n_{C_{1}}^{*}}\right)}^{1/\overset{*}{\underset{C_{1}}{\alpha }}}-\left[\Delta s\left(t\right)-{\left(\frac{a}{n_{C_{2}}^{*}}\right)}^{1/\overset{*}{\underset{C_{2}}{\alpha }}}\right]. \end{array}$$
(5) When *x*, *y* is (*x*3, *y*3), formula (23) is
  (23) $$\begin{array}{c} de\;J=\left(1-2x_{3}\right)\left[\Delta s\left(t\right)-{\left(\frac{a}{n_{C_{2}}^{*}}\right)}^{1/\overset{*}{\underset{C_{2}}{\alpha }}}-y_{3}k\left(1-e^{-b/a}\right)\Delta s\left(t\right)\right]+\left(1-2y_{3}\right)\left[kx_{3}\left(1-e^{-b/a}\right)\Delta s\left(t\right)-{\left(\frac{b}{n_{C_{1}}^{*}}\right)}^{1/\overset{*}{\underset{C_{1}}{\alpha }}}\right],\\ trJ=\left(1-2x_{3}\right)\left(1-2y_{3}\right)\left[\Delta s\left(t\right)-{\left(\frac{a}{n_{C_{2}}^{*}}\right)}^{1/\overset{*}{\underset{C_{2}}{\alpha }}}-y_{3}k\left(1-e^{-b/a}\right)\Delta s\left(t\right)\right]\times \left[kx_{3}\left(1-e^{-b/a}\right)\Delta s\left(t\right)-{\left(\frac{b}{n_{C_{1}}^{*}}\right)}^{1/\overset{*}{\underset{C_{1}}{\alpha }}}\right]\\ +k^{2}x_{3}y_{3}\left(1-x_{3}\right)\left(1-y_{3}\right){\left(1-e^{-b/a}\right)}^{2}{\left[\Delta s\left(t\right)\right]}^{2}. \end{array}$$

Based on the above five situations, when *de*  *J* > 0 and *trJ* < 0, there will be three parameter relationships, in which

Case I is
  (24) $$\begin{array}{c} {\left(\frac{b}{n_{C_{1}}^{*}}\right)}^{1/\overset{*}{\underset{C_{1}}{\alpha }}}>k\left(1-e^{-b/a}\right)\Delta s\left(t\right),\\ \Delta s\left(t\right)-{\left(\frac{a}{n_{C_{2}}^{*}}\right)}^{1/\overset{*}{\underset{C_{2}}{\alpha }}}>0. \end{array}$$
Case II is
  (25) $$\begin{array}{c} \Delta s\left(t\right)-{\left(\frac{a}{n_{C_{2}}^{*}}\right)}^{1/\overset{*}{\underset{2}{\alpha }}}>k\left(1-e^{-b/a}\right)\Delta s\left(t\right)>{\left(\frac{b}{n_{C_{1}}^{*}}\right)}^{1/\overset{*}{\underset{C_{1}}{\alpha }}}>0. \end{array}$$
Case III is
  (26) $$\begin{array}{c} \Delta s\left(t\right)-{\left(\frac{a}{n_{C_{2}}^{*}}\right)}^{1/\overset{*}{\underset{2}{\alpha }}}<0. \end{array}$$

According to the above three cases, the stability of five points in these cases is shown in Table 3.

### 3.3. Analysis of Evolutionary Path

When *n* = 3 and the income function is divided into three periods as the initial value *x*_1_, intermediate value *x*_2_=*αx*_1_+(1 − *α*)*x*_3_ with *α* ∈ [0,1], and target value *x*_3_, the paper believes that a stable point can be achieved during this period. To facilitate the calculation, the average industry return rate is assumed to be *r* = 10%. Income functions for managers and shareholders are, respectively, established, and strategies are adjusted as per the behavior of the other party [15, 16].

Managers:
(1) When *y*=0, assuming all shareholders do not supervise the earnings management, the income function of managers under the condition is as shown in
  (27) $$\begin{array}{c} R_{\left(x,0\right)}=\frac{R_{\left(x_{1},0\right)}}{{\left(1+r\right)}^{1}}+\frac{R_{\left(x_{2},0\right)}}{{\left(1+r\right)}^{2}}+\frac{R_{\left(x_{3},0\right)}}{r{\left(1+r\right)}^{3}}\\ =\left[\left(\frac{10}{11}+\frac{100}{121}\alpha \right)x_{1}+\left(\frac{10000}{1331}+\frac{100}{121}\alpha \right)x_{3}\right]\times \left[\Delta s\left(t\right)-{\left(\frac{a}{n_{C_{2}}^{*}}\right)}^{1/\overset{*}{\underset{C_{2}}{\alpha }}}\right]+\frac{12310}{1331}\left[\frac{m\times s_{n}\left(t\right)}{1-m}-d\right]. \end{array}$$
Take the partial derivative of *x*_1_, *x*_3_ to get the following function expressions, as shown in
  (28) $$\begin{array}{c} \frac{\partial R}{\partial x_{1}}=\left(\frac{10}{11}+\frac{100}{121}\alpha \right)\times \left[\Delta s\left(t\right)-{\left(\frac{a}{n_{C_{2}}^{*}}\right)}^{1/\overset{*}{\underset{C_{2}}{\alpha }}}\right], \end{array}$$
  (29) $$\begin{array}{c} \frac{\partial R}{\partial x_{3}}=\left(\frac{10000}{1331}+\frac{100}{121}\alpha \right)\times \left[\Delta s\left(t\right)-{\left(\frac{a}{n_{C_{2}}^{*}}\right)}^{1/\overset{*}{\underset{C_{2}}{\alpha }}}\right]. \end{array}$$
(2) When *y*=1, assuming all shareholders supervise the activity, the income function of managers under such condition will be as shown in
  (30) $$\begin{array}{c} R_{\left(x,1\right)}=\frac{R_{\left(x_{1},1\right)}}{{\left(1+r\right)}^{1}}+\frac{R_{\left(x_{2},1\right)}}{{\left(1+r\right)}^{2}}+\frac{R_{\left(x_{3},1\right)}}{r{\left(1+r\right)}^{3}}\\ =\left[\left(\frac{10}{11}+\frac{100}{121}\alpha x_{1}\right)+\left(\frac{10000}{1331}+\frac{100}{121}\left(1-\alpha \right)x_{3}\right)\right]\times \left[\Delta s\left(t\right)-{\left(\frac{a}{n_{C_{2}}^{*}}\right)}^{1/\overset{*}{\underset{C_{2}}{\alpha }}}-k\left(1-e^{-b/a}\right)\times \Delta s\left(t\right)\right]\\ +\frac{12310}{1331}\times \left[\frac{m\times s_{n}\left(t\right)}{1-m}-d\right]. \end{array}$$
Take the partial derivative of *x*_1_, *x*_3_ to get the following function expressions, as shown in
  (31) $$\begin{array}{c} \frac{\partial R}{\partial x_{1}}=\left(\frac{10}{11}+\frac{100}{121}\alpha \right)\times \left[\Delta s\left(t\right)-{\left(\frac{a}{n_{C_{2}}^{*}}\right)}^{1/\overset{*}{\underset{C_{2}}{\alpha }}}-k\left(1-e^{-b/a}\right)\Delta s\left(t\right)\right], \end{array}$$
  (32) $$\begin{array}{c} \frac{\partial R}{\partial x_{3}}=\left[\frac{1000}{1331}+\frac{100}{121}\left(1-\alpha \right)\right]\times \left[\Delta s\left(t\right)-{\left(\frac{a}{n_{C_{2}}^{*}}\right)}^{1/\overset{*}{\underset{C_{2}}{\alpha }}}-k\left(1-e^{-b/a}\right)\Delta s\left(t\right)\right]. \end{array}$$
Shareholders:
(3) When *x*=0, assuming all managers do not have earnings management, the income function of shareholders is as shown in
  (33) $$\begin{array}{c} R_{\left(0,y\right)}=\frac{R_{\left(0,y_{1}\right)}}{{\left(1+r\right)}^{1}}+\frac{R_{\left(0,y_{2}\right)}}{{\left(1+r\right)}^{2}}+\frac{R_{\left(0,y_{3}\right)}}{r{\left(1+r\right)}^{3}}\\ =\frac{12310}{1331}\times s_{n}\left(t\right)-\left[\left(\frac{10}{11}+\frac{100}{121}\alpha \right)y_{1}+\left(\frac{10000}{1331}+\frac{100}{121}\left(1-\alpha \right)\right)\right]\times {\left(\frac{b}{n_{C_{1}}^{*}}\right)}^{1/\overset{*}{\underset{C_{1}}{\alpha }}}. \end{array}$$
Take the partial derivative of *y*_1_, *y*_3_ , we get the following function expressions as shown in
  (34) $$\begin{array}{c} \frac{\partial R}{\partial y_{1}}=-\left(\frac{10}{11}+\frac{100}{121}\alpha \right)\times {\left(\frac{b}{n_{C_{1}}^{*}}\right)}^{1/\overset{*}{\underset{C_{1}}{\alpha }}}, \end{array}$$
  (35) $$\begin{array}{c} \frac{\partial R}{\partial y_{3}}=-\left[\frac{1000}{1331}+\frac{100}{121}\left(1-\alpha \right)\right]\times {\left(\frac{b}{n_{C_{1}}^{*}}\right)}^{1/\overset{*}{\underset{C_{1}}{\alpha }}}. \end{array}$$
(4) When *x*=1, assuming all managers have earnings management, the income function of shareholders is as shown in
  (36) $$\begin{array}{c} R_{\left(1,y\right)}=\frac{R_{\left(1,y_{1}\right)}}{{\left(1+r\right)}^{1}}+\frac{R_{\left(1,y_{2}\right)}}{{\left(1+r\right)}^{2}}+\frac{R_{\left(1,y_{3}\right)}}{r{\left(1+r\right)}^{3}}\\ =\frac{12310}{1331}\times \left[s_{n}\left(t\right)-\Delta s\left(t\right)\right]+\left\{\left(\frac{10}{11}+\frac{100}{121}\alpha \right)y_{1}+\left[\frac{10000}{1331}+\left(1-\alpha \right)y_{3}\right]\right\}\\ \times \left[-{\left(\frac{b}{n_{C_{1}}^{*}}\right)}^{1/\overset{*}{\underset{C_{1}}{\alpha }}}+k\left(1-e^{-b/a}\right)\times \Delta s\left(t\right)\right]. \end{array}$$
Take the partial derivative of *y*_1_, *y*_3_ , we get the following function expressions, as shown in
  (37) $$\begin{array}{c} \frac{\partial R}{\partial y_{1}}=\left(\frac{10}{11}+\frac{100}{121}\alpha \right)\times \left[-{\left(\frac{b}{n_{C_{1}}^{*}}\right)}^{1/\overset{*}{\underset{C_{1}}{\alpha }}}+k\left(1-e^{-b/a}\right)\times \Delta s\left(t\right)\right], \end{array}$$
  (38) $$\begin{array}{c} \frac{\partial R}{\partial y_{1}}=\left[\frac{10000}{1331}+\frac{100}{121}\left(1-\alpha \right)\right]\times \left[-{\left(\frac{b}{n_{C_{1}}^{*}}\right)}^{1/\overset{*}{\underset{C_{1}}{\alpha }}}+k\left(1-e^{-b/a}\right)\times \Delta s\left(t\right)\right]. \end{array}$$
The paper carries out a path analysis to the decision-making of managers and shareholders through a mathematical formula. Assuming the initial value of both parties of the game is either 0 or 1, the initial value of decision variables *x* and *y* of both parties is at any point from 0 to 1. Due to the inability of a mathematical formula in simulating decision behavior, the paper uses Python software to simulate the evolution of the decision-making behavior of both parties under different initial values. This section listed a stable point and an unstable point for illustration, assuming (1, 0) and (0, 1) are selected [17, 18].

The path of (1, 0): assume that none of the shareholders supervise the earnings management at the first stage, i.e., *y*=0, and the income function of managers is established as shown in formula (27). Then take the partial derivative of *x*_1_, *x*_3_, respectively, to get the function expressions as shown in formulas (28) and (29). It can be judged according to the formula:

When Δ*s*(*t*) − (*a*/*n*_*C*_2__^*∗*^)^1/*α*_*C*_2__^*∗*^^ > 0, formulas (28) and (29) are increasing functions, which means when *x*_3_=1, the income *R* is the maximum, referring to a situation where managers tend to choose earnings management.

The second stage: when shareholders find that managers have earnings management, the income function of shareholders is established as shown in formula (30), and then function expressions are gotten through taking the partial derivative of *y*_1_, *y*_3_, as shown in formulas (31) and (32). According to the formula:

When *k*(1 − *e*^−*b*/*a*^) × Δ*s*(*t*) < (*b*/*n*_*C*_1__^*∗*^)^1/*α*_*C*_1__^*∗*^^, formulas (37) and (38) are decreasing functions, which means when *y*=0, the income *R* is the maximum. Therefore, when the following conditions are met, Δ*s*(*t*) − (*a*/*n*_*C*_2__^*∗*^)^1/*α*_*C*_2__^*∗*^^ > 0, *k*(1 − *e*^−*b*/*a*^) × Δ*s*(*t*) < (*b*/*n*_*C*_1__^*∗*^)^1/*α*_*C*_1__^*∗*^^, the game between the two parties will eventually stabilize at (1, 0).

The path of (0, 1): assume that all shareholders choose supervision in the first stage, that is, *y*=1, and the income function of managers is established, as shown in the above formula (30). Then take the partial derivative of *x*_1_, *x*_3_, respectively, to get the function expressions, as shown in formulas (31) and (32). According to the formula:

When Δ*s*(*t*) − (*a*/*n*_*C*_2__^*∗*^)^1/*α*_*C*_2__^*∗*^^ < *k*(1 − *e*^−*b*/*a*^)Δ*s*(*t*), formulas (31) and (32) are decreasing functions, which means when *x*=0, the income *R* is the maximum. Under such circumstances, managers tend to choose no earnings management.

The second stage: when shareholders find that managers do not have earnings management, the income function of shareholders is established as shown in formula (33) and then take the partial derivative of *y*_1_, *y*_3_, respectively, to get the function expressions as shown in formulas (34) and (35). According to the formula:

Because the supervision cost of shareholders should be greater than 0, namely, (*b*/*n*_*C*_1__^*∗*^)^1/*α*_*C*_1__^*∗*^^ > 0, formulas (34) and (35) are decreasing functions, that is, when *y*=0, the income *R* is the maximum, which means the shareholders changed their behaviors so both parties are unable to be stable at the point (0, 0).

## 4. Analysis of Numerical Simulation

We analyze the game model of managers and shareholders in the second section. Since parameters in this paper lack specific data and cannot be replaced by any financial indicators, we use the Python software to assign values to each parameter for simulation, so as to show the evolution process of both parties of the game in the form of a graph and study the impact of change in each variable on the evolution process.

According to the theoretical model above, the relevant variables include counterfeiting efficiency *a*, supervision efficiency *b*, the proportion of managers' penalty amount *k*, shareholders' identification probability for earnings management income *β*, managers' additional income from earnings management Δ*s*(*t*), the strength of managers' counterfeiting ability *n*_*c*_2__^*∗*^, *α*_*c*_2__^*∗*^, and degree of shareholder supervision *n*_*c*_1__^*∗*^, *α*_*c*_1__^*∗*^.

The identification probability is *β*=1 − *e*^−*b*/*a*^, while assuming that managers' counterfeiting efficiency *a* is taken as 0, then the shareholders' identification probability for earnings management income *β* is equal to 1. Assuming that shareholders' supervision efficiency *b* is taken as 0, shareholders' identification probability for earnings management income *β* is equal to 0.

The paper assumes that the penalty amount is at least 0 and at most the doubled penalty on the basis of recovering the original amount, so the variation range of penalty proportion *k* is assumed to be 0–2.

The greater the value of *n*_*c*_2__^*∗*^, *α*_*c*_2__^*∗*^ representing the strength of managers' counterfeiting ability, the greater the effect of managers' unit counterfeiting cost. However, due to the difficulty of defining managers counterfeiting ability, it is assumed in this paper that managers' counterfeiting ability is a fixed value of an average level 1. Similarly, it is assumed that shareholders' supervision ability is also a fixed value of an average level 1.

### 4.1. Stability Test

Each variable is assigned a value under various parameter conditions. We assume that the initial time is 0 and the ending time is 5, while the horizontal axis represents the time *t* of the evolutionary game, and the vertical axis represents the decision variables *x*, *y* of both parties:

(1) Take the value of each parameter as
  (39) $$\begin{array}{c} {a=0,b=50,k=2,\Delta S}_{\left(t\right)}=20,\overset{*}{\underset{C_{1}}{n}}=1,\overset{*}{\underset{C_{1}}{\alpha }}=1,\overset{*}{\underset{C_{2}}{n}}=1,\overset{*}{\underset{C_{2}}{\alpha }}=1. \end{array}$$
The simulation results of variable relation that meets case I are shown in Figure 1 under different initial proportions of *x* and *y*:
Shareholders will choose not to supervise managers' earnings management when the supervision cost is greater than the supervision benefits. Managers' decision-making depends on the size of the net benefits generated by earnings management and the number of fines. In the case of (1, 0), the net income of earnings management is greater than 0, but it did not reflect the relationship between the net benefits and the fines. Enterprise managers will have earnings management when the net benefits of earnings management are greater than the fine amount. When the net benefits of earnings management are less than the fine, managers will not manage the earnings, but they will still observe shareholders' decisions. If there is no shareholder supervision, managers will eventually manage the earnings. The final stable point of evolution results of both parties is (1, 0); that is, managers choose to have earnings management while the shareholders do not supervise.
(2) Take the value of each parameter as
  (40) $$\begin{array}{c} {a=2,b=2,k=1,\Delta S}_{\left(t\right)}=20,\overset{*}{\underset{C_{1}}{n}}=1,\overset{*}{\underset{C_{1}}{\alpha }}=1,\overset{*}{\underset{C_{2}}{n}}=1,\overset{*}{\underset{C_{2}}{\alpha }}=1. \end{array}$$
The simulation results of variable relation that meets case II are shown in Figure 2 under different initial proportions of *x* and *y*:
Shareholders will supervise managers' behavior of earnings management when the supervision cost is less than the supervision benefits. Meanwhile, managers will manage the earnings when the net benefit of earnings management is greater than the fine amount. The final stable point of the game between managers and shareholders is (1, 1), which means managers choose to manage the earnings while the shareholders do not carry out supervision.
(3) Take the value of each parameter as
  (41) $$\begin{array}{c} {a=100,b=1,k=2,\Delta S}_{\left(t\right)}=50,\overset{*}{\underset{C_{1}}{n}}=1,\overset{*}{\underset{C_{1}}{\alpha }}=1,\overset{*}{\underset{C_{2}}{n}}=1,\overset{*}{\underset{C_{2}}{\alpha }}=1. \end{array}$$
The simulation results of variable relation that meets case II are shown in Figure 3 under different initial proportions of *x* and *y*:
Managers will not conduct earnings management when the activity generates little additional benefits. Shareholders' decision is up to the comparison of supervision cost and supervision benefits. Shareholders will supervise the earnings management when the cost is less than the benefits; otherwise, they will not supervise. After several games, however, shareholders may adjust their strategy from supervision to nonsupervision when they realize that managers do not conduct earnings management. The final stable point of the evolutionary game is (0, 0); that is, managers have no earnings management and shareholders do not supervise.

### 4.2. Sensitivity Test

To better describe and verify the impact of parameters on the evolutionary game, this section changes the value of each parameter according to the variable relationship of case I and analyzes the impact of changes in parameters on the evolutionary game. We select the evolutionary stable point (1, 0) to conduct a sensitivity test:

1. As other variables are unchanged, the value of Δ*s*(*t*) is changed to observe the impact of its change on the results of the evolutionary game. Assume that the value of managers' additional benefits Δ*s*(*t*) obtained from earnings management is, respectively, taken as 5 and 20, as shown in Figures 4 and 5, and the evolutionary process of Δ*s*(*t*)=20 is faster than that of Δ*s*(*t*)=5, that is, the increase in managers' additional benefits Δ*s*(*t*) obtained from earnings management can speed up the evolutionary game of both parties.
2. With other variables unchanged, we change the value of shareholders' supervision efficiency *b* and observe the impact caused by the change on the results of the evolutionary game. Assume that the value of *b* is, respectively, taken as 45 and 85, as shown in Figures 6 and 7, and the evolutionary process of *b*=85 is faster when *b*=45, so the increase in shareholders' supervision efficiency *b* can speed up the evolutionary game of both parties.
3. With other variables unchanged, we change the value of managers' counterfeiting efficiency *a* and observe the impact caused by the change on the results of the evolutionary game. Assume that the value of *a* is, respectively, taken as 2 and 10, as shown in Figures 8 and 9, and the evolutionary process of *a*=2 is faster than that of *a*=10, so the decrease in managers' counterfeiting efficiency *a* can speed up the evolutionary game of both parties.

## 5. Conclusions

The above analysis has clearly explained the results of the evolutionary game between the two parties. Based on the purpose of studying the behavior of enterprise managers' earnings management, the following suggestions are put forward for the interests of shareholders:

(i) Set stricter penalties for management fraud. Managers will manage earnings when the net benefits of earnings management are far greater than the risk of being punished by shareholders. The author suggests that corporations could build regulations framework to ensure managers undertake the losses incurred by supervision and then give up the strategy of earnings management. Meanwhile, the punishment to earnings management in current society is seldom convicted as criminal cases, and there are loopholes in current laws and regulations that give managers chances to commit fraud without being punished. It is obvious that managers will continue their financial fraud when the penalty amount is less than the net benefits of earnings management; thus, it seems meaningless for the punishment to managers. Therefore, the paper suggests strictly punishing the earnings management behavior that hurts shareholders' interests. The punishment to counterfeiters is not only up to the penalty amount but also closely related to the chances of identifying the wrong earnings management. Therefore, it is particularly important to improve the mechanism of identifying the illegal benefits generated during earnings management. Enterprises should know more about the various means of counterfeiting behaviors, to obtain clues on how managers grasp income through earnings management.
(ii) Improve enterprises' supervision system. Aiming at managers' earnings management, it is necessary for enterprises to strengthen their own supervision and improve shareholders' supervision efficiency. The supervision can be carried on from the following aspects:
Firstly, strengthen the external audit of enterprises. External audit performs a supervisory role in management fraud through surveys in the internal control of enterprises, thus gaining the general situation of enterprises before determining the scope of the audit. An external audit can also be helpful in understanding the authenticity and credibility of enterprises' financial reports as well as the deficiency of enterprises' internal control.
Secondly, enhance the internal audit, which can be carried on from the following aspects:
  1. Establish the perfect corporate governance structure with a functional internal audit department. For the past decades, companies are refining their governance structure where the internal audit serves as a vital component. It is an important task for enterprises to establish perfect corporate governance and improve the position of internal audits.
  2. Strengthen the legal governance and supervision of internal audits and enhance the status of internal audits. We should formulate laws and regulations concerning an internal audit, so as to strengthen the independence of internal audit and regulate the responsibilities and rights of internal auditors. Only by establishing a perfect legal system for an internal audit can we guarantee its independence, and the recognition of the internal audit's special position can fulfill the function it ought to have.
  3. Build a qualified team of internal auditors and improve their profession. Firstly, work ethics education is a necessity for internal auditors. Secondly, professional skill training is a must to maintain the competence of the team. Internal auditors must master the knowledge of accounting, auditing, law, taxation, foreign trade, finance, infrastructure construction, enterprise management, etc., and apply theory in daily practices to contribute themselves to enterprise development.
Thirdly, increase the number of external nonexecutive directors. Nonexecutive directors are usually working part-time for the enterprises, so they may not have a detailed and thorough understanding of the daily operation of the enterprises. Nonexecutive directors usually focus more on the market competitiveness and sustainability of enterprises. Moreover, nonexecutive directors receive a fixed salary which is not affected by corporate performance. Thus, having more nonexecutive directors on board will strengthen supervision on earnings management.

## Figures and Tables

**Figure 1:** The evolutionary result of (*x*, *y*) at the stable point (1, 0).

**Figure 2:** The evolutionary result of (*x*, *y*) at the stable point (1, 1).

**Figure 3:** The evolutionary result of (*x*, *y*) at the stable point (0, 0).

**Figure 4:** The evolutionary result of earnings management with an additional income of 5.

**Figure 5:** The evolutionary result of earnings management with an additional income of 20.

**Figure 6:** The evolutionary result of shareholder supervision efficiency of 45.

**Figure 7:** The evolutionary result of shareholder supervision efficiency of 85.

**Figure 8:** The evolutionary result of managers' fraud efficiency of 2.

**Figure 9:** The evolutionary result of managers' fraud efficiency of 10.

**Table 1:** Definition of variables.

Serial number	Variables	Definition
1	*s*_1_(*t*)	Income without managers earnings management
2	*s*_*n*_(*t*)	Normal income of shareholders
3	Δ*s*(*t*)	Additional income from earnings management by managers
4	*c*_2_(*t*)	Cost of managers' earnings management
5	*c*_1_(*t*)	Cost of shareholders' supervision
6	*f*(*t*)=*β* × *k* × Δ*s*(*t*)=(0 < *k* < 2)	Penalty amount of earnings management by managers (*β* is identification probability and *k* is penalty ratio)
7	*p*(*t*)=Δ*s*(*t*)	Loss of shareholders caused by managers' earnings management
8	*a*	Counterfeiting efficiency
9	*b*	Supervision efficiency
10	*d*	Effort cost that managers need to pay no matter whether they carry on earnings management or not

**Table 2:** Payment matrices.

		Player 2: shareholders	
		Supervision (*y*)	No supervision (1 − *y*)
Player 1: managers	Earnings management (*x*)	$\begin{array}{c} \left(ms_{n}\left(t\right)/1-m\right)+\Delta s\left(t\right)-c_{2}\left(t\right)-k\beta \Delta s\left(t\right)\\ -d \end{array}$ , *s*_*n*_(*t*) − *c*_1_(*t*)+*kβ*Δ*s*(*t*) − Δ*s*(*t*)	$\begin{array}{c} \left(ms_{n}\left(t\right)/1-m\right)+\Delta s\left(t\right)-c_{2}\left(t\right)\\ -d \end{array}$ , *s*_*n*_(*t*) − Δ*s*(*t*)
	No earnings management (1 − *x*)	(*ms*_*n*_(*t*)/1 − *m*) − *d*, *s*_*n*_(*t*) − *c*_1_(*t*)	(*ms*_*n*_(*t*)/1 − *m*) − *d*, *s*_*n*_(*t*)

**Table 3:** Stability results.

	Case I			Case II			Case III		
	Det	Tra	ESS	Det	Tra	ESS	Det	Tra	ESS
(0, 0)	Negative	Negative	Instable	Negative	Positive	Instable	Positive	Instable	ESS
(1, 0)	Positive	Negative	ESS	Negative	Negative	Instable	Positive	Positive	Instable
(1, 1)	Positive	Positive	Instable	Positive	Negative	ESS	Negative	Positive	Instable
(0, 1)	Negative	Positive	Instable	Positive	Positive	Instable	Negative	Negative	Instable
(*x*3, *y*3)	0		Saddle point	0		Saddle point	0		Saddle point

## Data Availability

The datasets used and/or analyzed during the current study are available from the corresponding author on reasonable request.
